# Liver and Kidney Surgical Anatomy to Verify the Effect of miR-221 on Organ Damage in Septic Rats

**DOI:** 10.1155/2022/2814431

**Published:** 2022-02-11

**Authors:** Bingtao Shi, Jialing Zhang, QiaoGe Chen

**Affiliations:** ^1^Department of Human Anatomy, Henan Medical College, Zhengzhou 451191, Henan, China; ^2^BasicMedical Experimental Center, Henan Medical College, Zhengzhou 451191, Henan, China

## Abstract

**Background:**

Related studies have shown that miR-221 has the ability to promote inflammatory response. This experiment mainly discusses the effect of miR-221 on acute liver and kidney injury in septic rats.

**Method:**

Thirty Sprague Dawley (SD) rats were randomly divided into a (1) control group, (2) sepsis group, (3) miR-221 overexpression group, (4) miR-221 inhibition group, (5) HECTD2 inhibition group, and (6) miR-221 overexpression + HECTD2 inhibition group. The sepsis rat model was prepared by cecal ligation and puncture (CLP). The expression levels of miR-221 and HECTD2 were detected by RT-qPCR. The levels of aspartate aminotransferase (AST) and alanine aminotransferase (ALT) in the liver were detected by the IFCC method. The levels of blood urea nitrogen (BUN) were detected by the creatine oxidase method. The levels of inflammatory factors were detected by ELISA. The apoptosis rate of liver and kidney cells was detected by flow cytometry. The expression of p65 protein was detected by western blotting.

**Result:**

RT-qPCR results showed that the expressions of miR-221 and HECTD2 were upregulated in septic rats (*P* < 0.05). Compared with group 1, the liver function index, kidney function index, liver and kidney apoptosis rate, serum inflammatory factor level, and p65 protein expression in each group were increased (*P* < 0.05). Compared with group 2, the liver function index, kidney function index, liver and kidney apoptosis rate, serum inflammatory factor level, and p65 protein expression in groups 4 and 5 were decreased (*P* < 0.05). Compared with group 2, the expression of HECTD2 was upregulated in group 3 (*P* < 0.05). Compared with group 3, the liver function index, renal function index, liver and kidney apoptosis rate, serum inflammatory factor level, and p65 protein expression were decreased in group 6 (*P* < 0.05).

**Conclusion:**

MiR-221 promotes the expression of HECTD2 in septic rats, and inhibition of miR-221 expression can reduce the degree of liver and kidney injury in septic rats.

## 1. Introduction

Sepsis is a common acute and critical disease in clinical practice. Infection by multiple pathogens including bacteria, fungi, and viruses can lead to sepsis. Patients often have systemic inflammatory response syndrome (SIRS) and even multiple organ failure [1]. Acute liver and kidney injury is a common severe complication of sepsis [2, 3], and its occurrence is closely related to the excessive activation of inflammatory factors. The large activation of inflammatory factors is the main mechanism of organ injury in patients with sepsis. Sepsis usually occurs in patients with a history of surgery or burns. Studies have shown that the incidence of sepsis is high, about 30% in intensive care patients, and is still increasing year by year [4].

microRNA is a kind of endogenous small noncoding RNA, which regulates gene expression after transcription and participates in various biochemical reactions. miR-221 is a member of the microRNA family, participates in the growth and development of organisms, and is abnormally expressed in a variety of cancer cells, playing an important role in the development of cancer [5–8]. In recent years, studies have also shown that miR-221 is related to the secretion of inflammatory factors, and many studies have confirmed that miR-221 may have proinflammatory effects [9, 10]. There are few studies on the role of miR-221 in acute liver and kidney injury in septic rats, so this study aims to discuss the role of miR-221 in the development of acute liver and kidney injury in septic rats.

## 2. Materials and Methods

### 2.1. Establishment and Grouping of Animal Models

Thirty male Sprague Dawley (SD) rats were purchased from Changsha Tianqin Biotechnology Co., Ltd., weighing (205 ± 20) *g*, and routinely fed for 7 days. Experimental rats were randomly divided into six groups: (1) control group, only the cecum was turned without ligation puncture; (2) sepsis group, cecum ligation and puncture (CLP) was performed; (3) miR-221 overexpression group, miR-221 mimic + CLP; (4) miR-221 inhibitor group, miR-221 inhibitor + CLP; (5) HECTD2 inhibition group, HECTD2siRNA + CLP; and (6) miR-221 mimic + HECTD2siRNA + CLP group. The CLP model was prepared according to the literature [11]. The rats in the model group were anesthetized with 10% phenobarbital sodium, and then, laparotomy was performed. After the cecum was removed, the cecum was ligated with No. 4 surgical silk thread at about 1/3 of the cecum root, and then, the distal cecum at the ligation site was gently pierced with a needle twice. The two perforations were about 3 cm apart, and then, the rice-sized feces were extruded from the perforation. The cecum was placed back into the abdominal cavity, and the incision was sutured. After successful sepsis modeling, miR-221 mimic, miR-221 inhibitor, HECTD2siRNA, and miR-221 mimic + HECTD2siRNA were injected into the tail of rats in the 3–6 group, respectively, with 5 *μ*L in each group. The peripheral blood was collected on the 4th day after continuous injection for 3 days. After the blood collection was completed, the rats were sacrificed by the cervical dislocation method, and the liver and kidney were dissected and sampled to preserve the tissues.

### 2.2. Quantitative Real-Time Polymerase Chain Reaction

Liver and kidney tissues were fully homogenized until the tissues were completely lysed. Total RNA was extracted by TRIzol reagent (from Thermo Fisher), and cDNA was synthesized according to the reverse transcription kit (from Invitrogen). The expression of miR-221 and HECTD2 in cells was detected by real-time quantitative PCR using cDNA as a template. The relative expression level was calculated by the 2^−ΔΔCt^ method. U6 was selected as the internal reference, and the primers used in the experiment (from Sangon Biotech) are shown in Table 1.

### 2.3. Detection of Liver and Kidney Function Indexes

Aspartate aminotransferase (AST) and alanine aminotransferase (ALT) were determined by the IFCC method, in strict accordance with the kit instructions (from Solar bio). The determination of serum creatinine (Cr) was carried out by the creatine oxidase method, and the determination of blood urea nitrogen (BUN) was carried out by the enzyme coupling rate method. Each index required about 100 *μ*l serum.

### 2.4. Enzyme-Linked Immunosorbent Assay

The serum of rats in each group was taken, and the levels of inflammatory cytokines IL-6, TNF-*α*, and IL-1*β* in peripheral blood were detected by using an ELISA kit (from eBioscience). The operation was carried out in strict accordance with the kit instructions.

### 2.5. Detection of Apoptosis Rate by Flow Cytometry

After the rats in each group were sacrificed, their liver and kidney tissues were crushed, digested with 0.25% trypsin (from Merck) for 3 h, and the cell suspension was obtained. A clean flow tube was taken and added with 300 *μ*L cell suspension and 5 *μ*L Annexin V-FITC (from ACROBiosystems) for 15 min in the dark. Then, 5 *μ*L PI staining solution and 200 *μ*L 1 *M*×Tris buffer were added. Apoptosis rate was detected by flow cytometry within 1 h.

### 2.6. Western Blotting

Each group of tissues were taken, cell lysate (from Beyotime, Shanghai, China) was added, and they were incubated on ice for 30 minutes. The protein in the cells was collected, and the total protein was quantified with the BCA protein detection kit. A 50 *μ*g protein sample was taken, and the protein was separated with 12% sodium lauryl sulfate-polyacrylamide gel, transferred to a nitrocellulose membrane (from Sigma), and blocked for 1 hour. Protein primary antibody (anti-p65, ab16502, Abcam, USA) was added and incubated overnight at 4°C. Secondary antibodies (from Abcam) were added at room temperature on the next day, incubated for 1 hour, and placed in the gel imaging system for exposure, and Quantity One software was used to analyze the gray value of protein bands.

### 2.7. Statistical Analysis

Statistical software SPSS 17.0 and GraphPad Prism 8.0.2 were used for statistical analysis of experimental data. Statistical data were analyzed with a *t*-test and then expressed as mean ± standard deviation. The count data were described by the utilization rate (%). *P* < 0.05represented that the difference had statistical significance.

## 3. Result

### 3.1. Expression of miR-221 and HECTD2 in Septic Rats

As shown in Figure 1, compared with the control group, the expression levels of miR-221 and HECTD2 in the sepsis group were significantly increased.

As shown in the figure, the levels of AST and ALT in the control group were the lowest and the levels of AST and ALT in the sepsis group were the highest. The levels of AST and ALT in the miR-221 inhibitor group were significantly lower than those in the sepsis group (*P* < 0.05, Figure 2(a)). The levels of Cr and BUN in the control group were the lowest, while those in the sepsis group were the highest. The levels of Cr and BUN in the miR-221 inhibitor group were significantly lower than those in the sepsis group (*P* < 0.05, Figure 2(b)). Flow cytometry results showed that the apoptosis rate of liver and kidney cells in the control group was the lowest and that in the sepsis group was the highest. The apoptosis rate of liver and kidney cells in the miR-221 inhibitor group was significantly lower than that in the sepsis group (*P* < 0.05, Figure 2(c)).

The levels of IL-6, TNF-*α*, and IL-1*β* in the control group were the lowest, and those in the sepsis group were the highest. The levels of IL-6, TNF-*α*, and IL-1*β* in the miR-221 inhibitor group were significantly lower than those in the sepsis group (*P* < 0.05, Figure 3).

The AST and ALT levels in the control group were the lowest, and those in the sepsis group were the highest. The AST and ALT levels in the HECTD2siRNA group were significantly lower than those in the sepsis group (*P* < 0.05, Figure 4(a)). The levels of Cr and BUN in the control group were the lowest, and those in sepsis group were the highest. The levels of Cr and BUN in the HECTD2siRNA group were significantly lower than those in the sepsis group (*P* < 0.05, Figure 4(b)). The results of flow cytometry showed that the apoptosis rate of liver and kidney cells in the control group was the lowest and that in the sepsis group was the highest. The apoptosis rate of liver and kidney cells in the HECTD2siRNA group was significantly lower than that in the sepsis group (*P* < 0.05, Figure 4(c)).

### 3.2. Effect of Inhibiting HECTD2 on Inflammatory Factor Levels in Septic Rats

The levels of IL-6, TNF-*α*, and IL-1*β* in the control group were the lowest, and those in the sepsis group were the highest. The levels of IL-6, TNF-*α*, and IL-1*β* in the HECTD2siRNA group were significantly lower than those in the sepsis group (*P* < 0.05, Figure 5).

### 3.3. miR-221 Promotes the Expression of HECTD2 in Septic Rats

Previous studies have confirmed the targeting relationship between miR-221 and HECTD2 [12], so this experiment is no longer repeated. RT-qPCR results showed that the expression of miR-221 in the miR-221 mimic group was significantly higher than that in the control group and sepsis group, indicating that the miR-221 mimic model was successfully constructed (Figure 6(a)). The expression of HECTD2 in the control group was the lowest, and the expression of HECTD2 in the miR-221 mimic group was significantly higher than that in the sepsis group (Figure 6(b)).

### 3.4. miR-221 Promotes Activation of the NF-*κ*B Pathway in Septic Rats

The expression level of p65 protein in the control group was the lowest, and that in the miR-221 mimic group was significantly higher than that in the sepsis group (^*∗*^*P* < 0.05 and ^*∗∗*^*P* < 0.05, Figure 7).

### 3.5. Inhibition of HECTD2 Expression Reverses the Effect of miR-221 on Liver and Kidney Injury in Septic Rats

The AST and ALT levels of rats in the control group were the lowest. Compared with the miR-221 mimic group, the AST and ALT levels were significantly decreased after HECTD2 inhibition (*P* < 0.05, Figure 8(a)). The levels of Cr and BUN in the control group were the lowest. Compared with the miR-221 mimic group, the levels of Cr and BUN after inhibiting HECTD2 were significantly decreased (*P* < 0.05, Figure 8(b)). The apoptosis rate of liver and kidney cells in the control group was the lowest. Compared with the miR-221 mimic group, the apoptosis rate of liver and kidney cells decreased significantly after inhibiting HECTD2 (*P* < 0.05, Figure 8(c)).

## 4. Discussion

Sepsis is a serious life-threatening disease, which not only has high morbidity and mortality but also requires a lot of medical resources [13]. Sepsis often occurs in major surgeries, large-area burns, poisoning, shock, and other diseases. Severe cases can progress to septic shock and multiple organ dysfunction syndrome, with high mortality [14]. When sepsis occurs, inflammatory cells in the body are activated, which can release a large number of inflammatory mediators, such as tumor necrosis factor, interleukin 1, and oxygen free radicals, causing serious damage to the tissues and organs of the body [15]. In this study, the classical CLP method was used to prepare a rat model of sepsis. It was found that the levels of AST, ALT, Cr, and BUN in the sepsis model rats were significantly increased after operation, and acute liver and kidney injury occurred. The levels of inflammatory factors and p65 protein expression were significantly increased. The results of flow cytometry showed that the apoptosis rate of liver and kidney cells in septic rats was significantly increased.

microRNAs (miRNAs) are a class of endogenous noncoding RNAs with 17–25 nucleotides in length, which are highly conserved in evolution. They widely exist in eukaryotic cells. They can participate in the posttranscriptional regulation of target genes by inducing their degradation or blocking the translation of target mRNAs through complementary binding with target mRNAs [16, 17] and play an important role in various biological activities [18, 19]. miR-221 is an oncogene-like miRNA that is abnormally expressed in a variety of cancer cells. In addition, studies have shown that miR-221 has the ability to regulate the expression of inflammation-related factors. Related studies have shown that miR-221 can regulate the inflammatory response of vascular endothelial cells by targeting adiponectin receptor 1 [20]. This study found that the expression of miR-221 in sepsis model rats was significantly increased, and inhibition of miR-221 expression could significantly reduce the liver and kidney function indexes and the apoptosis rate of liver and kidney cells in sepsis rats, suggesting that inhibition of miR-221 expression could reduce the degree of acute liver and kidney injury in sepsis rats.

HECTD2 is an E3 ubiquitin ligase. Related studies have shown that HECTD2 can ubiquitinize and degrade PIAS1, thereby aggravating the inflammatory response [21]. PIAS1 is a negative regulator of NF-*κ*B, and PIAS1 can bind to p65 protein to inhibit NF-*κ*B activity [22]. NF-*κ*B is an important factor regulating inflammation, immune response, and cell survival [23]. In the process of inflammation and tissue injury, NF-*κ*B regulates downstream inflammatory cytokines, which may be involved in the injury process. The NF-*κ*B signaling pathway is one of the key regulatory pathways of inflammatory response [24], and the changes in the expression of pathway-related genes such as CD14, MyD88, TNF-*α*, IL-1*β*, and IL-1R play an important role in the development of sepsis [25–28]. Our results showed that miR-221 can promote the expression of HECTD2 in septic rats, and overexpression of HECTD2 can partially reverse the promotion of miR-221 on liver and kidney injury in septic rats. The study has also indicated that HECTD2 is a downstream target of miR-221 and miR-221 could inhibit the expression of HECTD2 to boost the development of androgen independence in prostate cancer cells [12].

It is speculated that miR-221 can aggravate liver and kidney injury in septic rats by promoting the expression of HECTD2 and promoting the activation of NF-*κ*B.

In summary, our study confirmed that miR-221 had a promoting effect on acute liver and kidney injury in septic rats, which may be achieved by regulating the activity of the NF-*κ*B signaling pathway and the level of inflammatory factors. Inhibition of miR-221 may reduce the level of inflammatory factors and the activity of the NF-*κ*B signaling pathway, thereby reducing the degree of liver and kidney injury. However, there are many factors related to the regulation of sepsis acute organ injury, and this study still has certain limitations. The specific mechanism of miR-221 in the process of acute organ injury remains to be further studied.

## Figures and Tables

**Figure 1:** Expression levels of miR-221 and HECTD2. Inhibition of miR-221 expression attenuates acute organ injury in septic rats.

**Figure 2:** Effect of miR-221 on acute organ injury in septic rats. (a) Liver function indexes. (b) Kidney function index. (c) Apoptosis rate of liver and kidney cells. ^*∗*^*P* < 0.05,^*∗∗*^*P* < 0.05, and^*∗∗∗*^*P* < 0.05. Inhibition of miR-221 expression reduces inflammatory factor levels in septic rats.

**Figure 3:** Inflammatory factor levels. Inhibition of HECTD2 expression attenuates acute organ injury in septic rats.

**Figure 4:** Effect of inhibition of HECTD2 expression on acute organ injury in septic rats. (a) Liver function indexes. (b) Kidney function index. (c) Apoptosis rate of liver and kidney cells. ^*∗*^*P* < 0.05, ^*∗∗*^*P* < 0.05, and ^*∗∗∗*^*P* < 0.05.

**Figure 5:** Inflammatory factor levels.

**Figure 6:** Expression level of miR-221 and HECTD2.

**Figure 7:** miR-221 promoted the expression of p65 in the livers and kidneys of the rats. (A-B) The related expression of p65 in the livers and kidneys of the rats was detected with western blot. ^*∗*^*P* < 0.05 and ^*∗∗*^*P* < 0.05.

**Figure 8:** Inhibition of HECTD2 partially reverses miR-221 function. (a) Liver function indexes (AST and ALT). (b) Kidney function index (Cr and BUN). (c) Apoptosis rate of liver and kidney cells. ^*∗∗∗*^*P* < 0.05.

**Table 1:** Primer sequences of RT-qPCR.

Gene	Sequence
miR-221	F 5′-CCGCAGCTACATCTGGCTACTG-3′
	R 5′-GTGCAGGGTCCGAGGT-3′
HECTD2	F 5′-ATGAGTGAGGCGGTTCGGGT-3′
	R 5′-TGTACCATATGAAAAATAAAACCATCACTGATG-3′
U6	F 5′-GCTTCGGCAGCACATATACTAAAAT-3′
	R 5′-CGCTTCACGAATTTGCGTGTCAT-3′

## Data Availability

Data supporting the findings of this study are available on reasonable request from the corresponding author.
